# Breast Tumor Detection Using Robust and Efficient Machine Learning and Convolutional Neural Network Approaches

**DOI:** 10.1155/2022/6333573

**Published:** 2022-06-07

**Authors:** Mohammad Monirujjaman Khan, Tahia Tazin, Mohammad Zunaid Hussain, Monira Mostakim, Taeefur Rehman, Samender Singh, Vaishali Gupta, Othman Alomeir

**Affiliations:** ^1^Department of Electrical and Computer Engineering, North South University, Bashundhara R/A, Dhaka 1229, Bangladesh; ^2^IT Department, GLBajaj ITM, Greater Nodia, India; ^3^Computer Science & Engineering, Galgotias University, Greater Nodia, India; ^4^Department of Pharmacy Practice, College of Pharmacy, Shaqra University, Shaqra, Saudi Arabia

## Abstract

Breast cancer develops when cells in the breast expand and divide uncontrollably, resulting in a lump of tissue known as a tumor. This lump of tissue is called a tumor. After skin cancer, breast cancer is the second most common cancer among women. It is more common in women over the age of 50. Men may also acquire breast cancer, albeit it is uncommon. Each year, approximately 2,600 men in the United States are diagnosed with breast cancer, accounting for less than 1% of all cases. Transgender women are more likely than cisgender men to acquire breast cancer. Additionally, transgender males are less likely than cisgender women to acquire breast cancer. Breast cancer is more common in women over the age of 50, although it can affect anyone at any age. Early detection of a breast tumor may significantly lower the risk of developing breast cancer. A public dataset of breast tumor features was used instead to build models for identifying breast tumors through machine learning and deep learning. Prediction models were built using logistic regression (LR), decision tree (DT), random forest (RF), voting classifier (VC), support vector machine (SVM), and a proprietary convolutional neural network (CNN). These models were used to find critical prognostic indicators linked to breast cancer. The proposed network performs far better, with an average accuracy of 99%. This study has six types of models: LR, RF, SVM, VC, DT, and a custom CNN model. They all had 96% to 99% accuracy in this study. CNN, LR, RF, SVM, VC, and DT achieved 99%, 96%, 98%, 97%, 97%, and 96% F1 score, respectively. There were many machine learning algorithms used in this study that were very accurate, which means that these techniques could be used as alternative prognostic tools in breast tumor detection studies in Asia.

## 1. Introduction

Breast tumors (bosom disease) are quite possibly the most widely recognized tumors in women. As per a 2013 WHO study, “it is projected that more than 508,000 ladies passed away all around the world in 2011 because of bosom disease” [1]. Breast malignant growth is treatable and preventable in its early phases. Nonetheless, many women are diagnosed with malignant growth after it has progressed beyond the point of no return. Bosom disease is a dangerous growth that creates in the bosom cells greasy tissues or sinewy connective tissues. Bosom malignant growth cancers frequently decay and spread rapidly over time, eventually resulting in death [2]. Despite the fact that it is more prevalent in women, it might happen in men also. Bosom malignant growth chances may also be increased by a few factors, such as age and family ancestry. Bosom disease cancers are separated into harmless and dangerous subtypes [3].

A harmless growth represents no danger to the human body, and causing mortality in humans is exceptionally surprising. This type of cancer is confined and has a limited development rate. A threatening growth, then, is more destructive and might be lethal to individuals. This type of growth occurs quickly because of atypical cell multiplication. Obtrusive ductal carcinoma, ductal carcinoma *in situ*, and intrusive lobular carcinoma are the three types of malignant development found in the breast. Ductal carcinoma *in situ*, the first stage of bosom malignant development, is curable. The most pervasive sort of bosom disease is intrusive ductal carcinoma, which starts in the milk conduit. Intrusive lobular carcinomas can swiftly spread to lymph hubs and other parts of the body. It begins in the lobule of the bosom. Every year, around 1,000,000 women worldwide are determined to have bosom malignant growth. Endurance rates might be high in the beginning phases, but as of now, the five-year endurance rate is 81%. However, only 35% of ladies determined to have late-stage or metastatic bosom disease endure five years. Turkki et al. [4] claim that prognostic assessment can be done without prior knowledge of the histology of bosom malignant development. Utilizing five AI characterization strategies and one special CNN model, this study presents another AI and profound learning grouping strategy for bosom growth arrangement. The accompanying order procedures were inspected for execution: strategic relapse, arbitrary woods, support vector machine, casting a ballot classifier, choice tree, and custom CNN model. On the freely accessible breast tumor features dataset, the proposed approach is tested for execution. Numerous researchers have focused on the handiness of AI and profound learning in medical care to further develop therapy quality and wellbeing [5–12]. Bejnordi et al. [9] utilized a profound learning framework to identify bosom disease cancers and afterward contrasted the outcomes with pathologists' analyses. As indicated by the discoveries, programmed location using a profound learning framework outperformed human conclusion. Khan et al. [13] utilized motion to figure out how to combine highlights gotten from GoogleNet, VGGNet, and ResNet. Utilizing information mining strategies, Wang and Yoon [14] recommended an exceptional methodology for bosom malignant growth expectations. They formulated a technique for anticipating bosom malignant growth in light of the clinical information of patients. The approach was tested on two widely used public datasets: the Wisconsin Breast Cancer Database (WBCD) and the Wisconsin Diagnostic Breast Cancer Database (WDBCD) (WDBC). SVMs, eight learning models, ANNs, Naive Bayes grouping, and the AdaBoost Tree were all thoroughly tested. They thought of a method for eliminating highlights that pre-owned head part investigation and different information mining strategies, as well as a method for utilizing different models, similar to k-mean. Nguyen et al. [15] employed both administered and solo order models for bosom cancer orders. For example, to include determination, they suggested joining scaling and head part investigation. They showed that the best expectation model is a group casting a ballot. Following element choice, the information was utilized to test and prepare numerous classification models. Out of all the models used for the expectation, only four, troupe casting a ballot classifier, strategic relapse (LR), SVM, and AdaBoost, performed better, with an accuracy of around 90% in terms of model accuracy and review, Area Under the Receiver Operating Characteristics (AUC-ROC), F1 measure, and computational time. Choice trees (DTs), fake brain organizations (ANNs), and support vector machines were used by Ahmed et al. [16] (SVMs). SVMs [17] outflank different classifiers on the WBCD, as evidenced by the execution of several approaches. The DT, ANN, and SVMs were all 93.6%, 94.7%, and 95.7%accurate, respectively. For the evaluation, they performed a 10-overlay cross-approval. In their study, Mandal et al. [18] used LR, NB, and DTs. They additionally checked every classifier's fleeting intricacy. With the most elevated precision, LR outperforms different classifiers. Borges et al. [19] compared Bayesian and DT presentations and found that Bayesian organizations outflanked DT with 97.80% precision. Chaurasia and colleagues [20] utilized the WBCD dataset to break down the results and shaped an expectation model utilizing preprocessing, information choice, and information change. With an arrangement exactness of 97.36%, they discovered that Nave Bayes beat other models. the radial basis function (RBF) network and J48 had 96.77%and 93.41% arrangement exactness, respectively. To predict bosom malignant growth, Kumar et al. [21] used AdaBoost, J-Rip, LR, apathetic student, choice table, IBK, J48, languid K-star, multiclass classifier, multi-facet perceptron, arbitrary woodland, Nave Bayes, and irregular tree. That's what they guaranteed, except for Nave Bayes characterization, the calculations generally performed better compared to 94% of the time, and that apathetic and tree orders outscored other arrangement techniques by close to 100%. In spite of the fact that outfit learning works on the presentation of a base student, it lessens the predisposition or fluctuation, as indicated by Lee et al. [22]. Abdar and Makarenkov [23] introduced CWV-BANNSVM, a unique characterization method that coordinates a boosting artificial neural network (BANN) with two SVMs to optimize WBCD execution. Alam et al. [24] presented a novel and powerful group learning method to naturally recognize the quantity of brain organizations and their plans, rather than standard outfit learning. For each brain organization, different preparation sets are utilized, guaranteeing further development gains from all of the preparation information tests. Utilizing a steady preparation strategy, the recommended DEL is prepared various times to decide the ideal upsides of the learning rate boundary and the connection strength boundary. Improvement is feasible when using the troupe supporting methods, according to Osman and Aljahdali [25]. The technique was joined with a radial basis function brain network calculation, which further developed execution for the WBCD dataset to 98.4% accuracy. The greater part of the distributed examination evaluates the proposed strategy's presentation as far as “exactness.” Precision improves when the number of genuine up-sides (TPs) and genuine negatives (TNs) is greater than the number of bogus up-sides (FPs) and misleading negatives (FNs) (FNs). Accuracy and review, regardless of correctness, are essential for execution detailing regards to clinical findings; computerized reasoning frameworks ought to focus on bogus negatives (review) above misleading upsides (precision), since missing an illness could have disastrous repercussions for patients. Therefore, it is basic to evaluate execution utilizing f-gauges that focus on review over precision. Early detection of breast cancer may help with adjustment, which is not always possible. To forestall significant mischief, we will have to have a superior handle on a couple of bosom growth-related markers. The primary inspiration of this examination is to foresee bosom malignant growth by assessing information from those files, utilizing five AI and one profound learning characterization system to estimate the sickness, and then choosing the methodology with the best precision rate. Utilizing an assortment of approaches, most of the exams dissected had the option to achieve over 90% exactness. The principal objective of this study is to foster an AI and profound learning-based approach that can identify bosom cancers at an early phase. Our study makes a substantial addition in that we used a variety of well-known AI and deep learning methodologies to get our results. Then again, AI and convolutional brain networks are man-made brainpower methods that take into account thorough testing of different datasets to reveal already obscure examples and connections. AI strategies have been utilized to explore bosom growth expectations, and they show guarantee regarding early identification and anticipation. The current review, then again, offers another CNN engineering and AI strategy that will build on the precision of the bosom growth order. The new CNN model and AI calculations will actually want to eliminate how much manual work is currently done in clinical practice. Furthermore, the intriguing aspect of this study is that the recommended strategy uses fewer registered assets and accurately identifies bosom malignant growths 99% of the time. The remainder of the paper is structured as follows: Section 2 describes the suggested technique, which is followed by the experimentation and discussion of the results of Section 3.  Section 4 brings the work to a close by suggesting some future research directions for breast cancer tumor categorization.

## 2. Methods and Materials

The data was obtained from publicly available online sources. After separating the training and test sets, the recommended approach begins by loading and extracting data from raw datasets, followed by preprocessing and feature selection procedures. The framework of the suggested strategy, as well as hyper-parameter setup, regularization techniques, and an optimization algorithm are then presented. Finally, calculations for network training and performance are provided. Breast cancer and healthy data are classified using the CNN model, which was developed by Google Colab.

### 2.1. Dataset Description and Preprocessing

The breast tumor features dataset has been used in this research [26]. This dataset has 683 rows and 11 features of breast tumors. In the target column (class), 444 data indicate healthy breasts and 239 data indicate breast tumors. The first and last five rows of the dataset are shown in Figure 1.

Before model improvement, data preprocessing is necessary to remove unwanted noise and abnormalities from the dataset that could cause the model to deviate from the anticipated preparation set. This progression centers around eliminating any hindrances to the model's productivity. When the data has been gathered, it should be purified and prepared for model creation. From that point on, the dataset is examined for invalid qualities. Be that as it may, there are no invalid qualities in this dataset. As seen in Figure 2, this dataset contains no missing data.

The numbers “false” and “0” demonstrate that no invalid qualities are available. The following stage is to foster the model, subsequent to completing information readiness and dealing with the imbalanced dataset. The “example code number” segment has been eliminated in light of the fact that this section is unimportant to the objective section. To work on the assignment's exactness and effectiveness, the information is isolated into preparing and testing segments, with a preparation to testing proportion of 80/20. Following the separation of the model, it is prepared by utilizing a variety of groupings.

### 2.2. Feature Selection

Clump Thickness, Uniformity of Cell Size, Uniformity of Cell Shape, Marginal Adhesion, Single Epithelial Cell Size, Bare Nuclei, Bland Chromatin, Normal Nucleoli, and Mitoses all showed positive correlation coefficients between characteristics and the class label in the heat map. The feature correlation value and heatmap are shown in Figures 3 and 4, respectively.

All the features are positively correlated with the target column except “sample code number.” It is negatively correlated with the class column. For this reason, this column has been removed from the training and testing part.

Clump Thickness, Uniformity of Cell Size, Uniformity of Cell Shape, Marginal Adhesion, Single Epithelial Cell Size, Bare Nuclei, Bland Chromatin, Normal Nucleoli, and Mitosesis 71%, 82%, 82%, 71%, 69%, 82%, 76%, 72%, and 42% positively correlated with the target column (class).

### 2.3. Proposed Method

Figure 5 shows the proposed machine learning method block diagram.

Once the data has been analyzed, it is now accessible for model creation. Model creation requires a preprocessed dataset as well as machine learning algorithms. LR, DT classification, RF classification, SVM classifier, and voting classifier are some of the methods used. The accuracy score, precision score, recall score, and F1 score are the accuracy measurements. After five distinct machine learning models have been constructed, they are utilized to evaluate them.

The LR classification method [27] is a popular choice for modeling binary classifications. Linearly combining the input characteristics is thought to make one of the two output classes more likely than the other one [28]. This classification model's logistic equation is

(1) $$\begin{array}{c} Z_{a}=\ln\left(P_{a}÷\left(1-P_{a}\right)\right), \end{array}$$

where *P* denotes the probability of the incidence of event *a*

A support vector machine, or SVM, is a machine learning technique for dividing data into two categories. Support vector machines, also known as support vector classification, are guided and linear machine learning techniques that are most typically used to solve classification issues. Support vector regression (SVR) is a subset of support vector machines (SVM) that uses the same concepts to solve regression problems. The kernel approach, which essentially aids in resolving the non-linearity of the solution in a very straightforward way, is the most frequently utilized and useful feature of SVM.

One of the most frequently used supervised machine learning techniques for a graphical depiction of all potential answers is the random decision tree [29]. The options are straightforward and are dependent on specific conditions. It identifies and prioritizes the key traits that facilitate categorization. Only the qualities that gain the most information are chosen (IK). The following is how IK is defined:

(2) $$\begin{array}{c} \text{IK}=N\left(\text{Parent}-\text{Node}\right)-\text{Average }N\left(\text{Sub}-\text{Nodes}\right). \end{array}$$

RF classification was utilized as the characterization calculation. RFs are comprised of various separate choice trees that were each prepared based on an irregular example of information. These trees are made during the preparation interaction, and the results of the choice trees are gathered. This calculation's outcome is still up in the air by a cycle known as “casting a ballot.” This procedure requires each DT to decide in favor of one of two result classes (for this situation, “cancer” or “solid”). The RF technique, which picks the class with the best votes, decides the last estimate. In ensemble classification, majority-based voting [30] is extensively utilized. It is also known as plurality voting. After utilizing the three classification methods outlined above, the approaches discussed here [31] use a majority-based voting mechanism to increase classification performance.

For each test case, the model classification results are generated, and the ultimate outcome is forecasted based on the majority of the findings.

The majority vote of each classifier *P* predicts the class label *R* in majority voting.

(3) $$\begin{array}{c} R=\text{mode}\left\{P_{1}\left(x\right),P_{2}\left(x\right),\ldots ,P_{n}\left(x\right)\right\}. \end{array}$$

#### 2.3.1. Architecture of Convolutional Neural Network (CNN)

A CNN is a complex feed-forward brain network that works by stacking different secret layers on top of each other in response to a specific request. Convolutional neural networks might learn various levels of highlights on account of their consecutive development. More often than not, convolutional layers are trailed by initiation layers. Some of them are trailed by pooling layers.  Figure 6 shows the CNN architecture.

The convolutional layer is the most important component of a CNN. A convolutional layer may be seen as a series of little square templates called convolutional kernels that glide over the data looking for patterns. The kernel returns a big positive number when that section of the input fits the kernel's pattern, and zero or a lesser value when there is no match.

The suggested research employs a one-dimensional convolutional neural network (Conv1D). Each point in the input data is determined by a kernel calculation in the convolutional layer. As described in the design, dense input of 128 neurons is provided to the algorithm's input layer. Rectified Linear Unit is the work's activation layer (Relu). The first hidden layer receives pool size one, whereas the second hidden layer receives Maxpooling with pool size two. Problems involving noise and sparse gradients are solved using the Adam optimizer. For error computations, the mean-squared error is employed, and the accuracy metric is assessed.

### 2.4. Performance Matrix

On a confusion matrix, the system presented actual and anticipated values. The confusion matrix represents the forecast results of a classification model. The following precision, sensitivity, specificity, and accuracy values have been determined:

(4) $$\begin{array}{c} \text{Precision}=\frac{\text{TP}}{\text{TP}+\text{FP}}\text{,}\\ \text{Recall}=\frac{\text{TP}}{\text{TP}+\text{FN}}\text{,}\\ \text{Accuracy}=\frac{\text{TP}+\text{TN}}{\text{TP}+\text{FP}+\text{TN}+\text{FN}}\text{,}\\ \text{F}1=2*\frac{\text{Precision}*\text{Recall}}{\text{Precision}+\text{Recall}}. \end{array}$$

The term “True Positive” represents the number of cases that are expected to be favorable and actually occur (TP). The percentage of predicted negative situations that are also true negatives is referred to as True Negative (TN). A False Negative (FN) is a word used to describe the number of projected negative occurrences that come out to be positive, also known as a type two error. The number of expected positive examples that turn out to be negative is known as a “False Positive” (FP).

## 3. Result and Analysis

The proposed work uses the Keras and TensorFlow packages in Python 3.6, as well as other required libraries like matplotlib and pandas. For the experiment, CNN, a deep learning algorithm, was used. According to the results of the experiment, breast tumor prediction using the CNN algorithm had a validation accuracy of 99%.

### 3.1. CNN Model Accuracy and Loss

The training and validation accuracy graph, as well as the training and validation loss graph, are shown in Figures 7 and 8.

We divided the dataset into three components for the CNN model: training, validation, and testing. We used 77.31% of the data for training, 12.59% for validation, and the remaining 10.10% for verification. The model was trained using a learning rate of 0.0001, 128 batch sizes, and 50 epochs. With each epoch, the model's performance increases. The performance increases considerably in the first few epochs. The validation accuracy was 95.35%, and the training accuracy was 98.30%. Following that, we ran a test dataset through the model and obtained a 99% F1 score.

The CNN model's training and validation losses are shown in Figure 8. The validation loss was 6.72%, while the training loss was 4.89%. Because the training accuracy is larger than the validation accuracy and the validation loss is greater than the training loss, this model does not have an overfitting problem.  Figure 9 shows the classification report of the CNN model.

CNN achieved 98.6% test accuracy. The training accuracy was 98.30%for the CNN model. Here, 0 denotes non-tumor data and 1 denotes tumor data. The precision was 98% for non-tumor data and 99% for tumor data. Also, the recall was 100% for non-tumor data and 96% for tumor data. And for tumor and non-tumor data f1-score was 99% and 98%, respectively. The CNN model's confusion matrix is shown in Figure 10.

The model's computed performance is displayed alongside the anticipated result in the confusion matrix. There were 68 correct predictions and 1 incorrect ones.

### 3.2. Machine Learning Model Accuracy

#### 3.2.1. Logistic Regression

Figure 11 shows the classification result of the logistic regression model.

LR achieved 96% test accuracy. The training accuracy was 98% for the logistic regression model. Here, 2 denotes tumor and 4 denotes non-tumor data. The precision was 93% for tumor data and 99% for non-tumor data. Also, the recall was 99% for tumor data and 94% for non-tumor data. And for both tumor and non-tumor data f1-score was 96%.  Figure 12 depicts the logistic regression model's confusion matrix.

Label 1 indicates a “tumor” and Label 0 indicates “non-tumor” data. The row corresponds to the actual level, while the column corresponds to the anticipated label. This model correctly predicted 171 data and incorrectly predicted 7 data.

#### 3.2.2. Random Forest

The classification result of the random forest model is shown in Figure 13.

Random forest achieved the highest test accuracy, 98%. The training accuracy was 100% for the RF model. Here, 2 denotes tumor and 4 denotes non-tumor data. The precision was 98% for tumor data and 99% for non-tumor data. Also, the recall was 99% for tumor data and 98% for non-tumor data. For both tumor and non-tumor data, f1-score was 98%.  Figure 14 shows the confusion matrix of the random forest model.

With 300 estimators, the random forest model predicted 175 data correctly. This is the highest number of correct predictions in this research. Also, this model incorrectly predicted only three data. This is the lowest incorrect prediction rate.

#### 3.2.3. Support Vector Machine

Figure 15 shows the support vector machine classifier's result.

SVM achieved the second-highest test accuracy, 97%. The training accuracy was 100% for the SVM model. The precision was 94% for tumor data and 99% for non-tumor data. Also, the recall was 99% for tumor data and 95% for non-tumor data. And for both tumor and non-tumor data f1-score was 97%. The SVM model's confusion matrix is shown in Figure 16.

After fine-tuning, the SVM model predicted 172 data correctly. This is the second-highest number of correct predictions in this research. Also, this model incorrectly predicted only six data. The number of correct predictions is less than the RF model's prediction, and the number of incorrect predictions is greater than the RF model's prediction.

#### 3.2.4. Voting Classifier

Figure 17 shows the voting classifier's model result.

VC achieved the second-highest test accuracy as an SVM classifier, at 97%. The training accuracy was 100% for the VC model. The precision was 95% for tumor data and 99% for non-tumor data. Also, the recall was 99% for tumor data and 96% for non-tumor data. And for both tumor and non-tumor data f1-score was 97%.  Figure 18 shows the confusion matrix of the voting classifier model.

Without fine-tuning, the voting classifier model predicted 173 data correctly. Also, this model incorrectly predicted only five data. In this case, the number of correct predictions is less than the RF model's prediction, and the number of incorrect predictions is also greater than the RF model's prediction.

#### 3.2.5. Decision Tree Classifier

The classification result of the decision tree classifier is shown in Figure 19.

The decision tree achieved the lowest test accuracy of 96%. The training accuracy was 99% for the DT model. The precision was 94% for tumor data and 98% for non-tumor data. Also, the recall was 98% for tumor data and 95% for non-tumor data. And for both tumor and non-tumor data f1-score was 96%.  Figure 20 shows the confusion matrix of the voting classifier model.

After fine-tuning, the decision tree classifier model predicted 171 data correctly. Also, this model incorrectly predicted only seven data. In this case, the number of correct predictions is lower than the above four algorithms, and for this reason, this model achieved the lowest accuracy in this research.

### 3.3. Comparison of Result

This study combined both machine learning and deep learning approaches in order to identify a breast tumor in its early stages. The suggested CNN and machine learning models are compared to the previous research in Table 1. With 300 estimators, the recommended random forest model was 98% accurate.

By fine-tuning the random forest algorithm, this study achieved 98% accuracy. Using the same strategy, Ref. [28] achieved an accuracy of 93.50%. Furthermore, using the SVM classifier, this work achieved 97% accuracy, whereas Ref. [29] achieved 89.20% accuracy. This article obtained 99% test accuracy using the CNN model, but Ref. [25] reached 97% accuracy using a different neural network, which is somewhat better than this study. The accuracy rate of the models utilized in this study is significantly higher than that of earlier research, implying that they are more dependable than previous models.

## 4. Conclusion

Breast cancer provides a unique context for medical diagnosis by taking into account the patients' condition and treatment response. Breast cancer detection has been considerably helped by machine learning. Despite technological advancements, accurate detection and monitoring of breast cancer remains a challenge. The biological, social, and demographic streams of data must all be combined to improve prediction models. To propose both machine learning and deep learning for classification, we examined the performance of basic logistic regression learning, random forest, decision tree, and support vector machine learning with sequential minimum optimization, voting classifier, and convolutional neural network. The performance of these six classifiers was assessed using a variety of performance measures, including accuracy, precision, recall, and F1 score. In this study, a custom CNN model achieved 99% F1 score. On the other hand, LR, RF, SVM, VC, and DT achieved 96%, 98%, 97%, 97%, and 96% F1 score, respectively. We plan to test multiple feature selection method in the next to determine which one may assist us uncover the smallest group of traits that can reliably categorize breast cancer as benign or malignant. Researchers can compare the results of several weighted voting methods, such as basic weighted voting, rescaled weighted voting, best-worst weighted voting, and quadratic best-worst weighted voting, rather than utilizing an unweighted voting mechanism. Other breast cancer classification datasets could be used to test and improve the performance of the proposed method. This latest results can be used to classify breast tumors using images as a starting point.

## Figures and Tables

**Figure 1:** The first and last five rows of the dataset.

**Figure 2:** Zero missing value.

**Figure 3:** Feature correlation matrix.

**Figure 4:** Feature correlation matrix-heatmap.

**Figure 5:** Proposed machine learning method system block diagram.

**Figure 6:** Architecture of a CNN.

**Figure 7:** CNN model training and validation accuracy.

**Figure 8:** Training and validation loss for CNN model.

**Figure 9:** Classification result of CNN model.

**Figure 10:** Confusion matrix of CNN.

**Figure 11:** Classification result of logistic regression model.

**Figure 12:** Confusion Matrix of LR model.

**Figure 13:** RF classification result.

**Figure 14:** RF confusion matrix.

**Figure 15:** SVM classification result.

**Figure 16:** SVM confusion matrix.

**Figure 17:** VC classification result.

**Figure 18:** VC confusion matrix.

**Figure 19:** DT classification result.

**Figure 20:** DT confusion matrix.

**Table 1:** Result comparison.

This Research (Algorithm Name)	Accuracy (%)	Reference Paper (Model Name)	Accuracy (%)
Random forest	98	Ref. [28] Random Forest	93.50
Support vector machine	97	Ref. [29] Support Vector Machine	89.20
Voting classifier	97	Ref. [30] Naïve Bayes	74.24
Convolutional neural network	99	Ref. [25] Neural Network	97.00

## Data Availability

The data utilized to support these research findings are accessible online at https://www.kaggle.com/ayushish12/breast-tumor-features.
